The article "An Improved Epidemiological Model for the Underprivileged People in the Contemporary Pandemics" was published in 2022. Journal: Biomed Res Int.

# An Improved Epidemiological Model for the Underprivileged People in the Contemporary Pandemics

**DOI:** 10.1155/2022/7890821

**Published:** 2022-10-11

**Authors:** Mahtab Uddin, Shafayat Bin Shabbir Mugdha, Tamanna Shermin, Kawsar Newaz Chowdhury

**Affiliations:** ^1^Institute of Natural Sciences, United International University, Dhaka 1212, Bangladesh; ^2^Department of Computer Science & Engineering, United International University, Dhaka 1212, Bangladesh

## Abstract

In this work, we introduce an improved form of the basic SEIRD model based on Python simulation for the troublesome people who are oblivious about the contemporary pandemics due to diverse social impediments, especially those economically underprivileged. In the extant epidemiological models, some unorthodox issues are yet to be considered, such as poverty, illiteracy, and carelessness towards health issues, significantly influencing the data modeling. Our focus is to overcome these issues by adding two more branches, for instance, uncovered and apathetic people, which significantly influence the practical purposes. For the data simulation, we have used the Python-based algorithm that trains the desired system based on a set of real-time data with the proposed model and provides predicted data with a certain level of accuracy. Comparative discussions, statistical error analysis, and correlation-regression analysis have been introduced to validate the proposed epidemiological model. To show the numerical evidence, the investigation comprised the figurative and tabular modes for both real-time and predicted data. Finally, we discussed some concluding remarks based on our findings.

## 1. Introduction

To investigate the future of a system, we need a proper representation of that system. However, often we find it difficult to infer how the system functions as a whole. Mathematical modeling provides a framework for conceptualizing our ideas through some equations, which assist in developing new hypotheses for future testing [1]. It is used in various settings, including disease mechanism analysis, biomedical systems, and government policymaking. William Ogilvy Kermack and Anderson Gray McKendrick are the introducers of mathematical modeling into the field of epidemiology [2]. It immensely aids in the quantification of potential infectious disease control and mitigation techniques. It provides a crude general behavior of an epidemic as addressed by epidemic curves, allowing predictions about the epidemic's endurance, magnitude in the population, and evaluation of components that influence transmission dynamics and thus the number of cases [3].

Mathematical modeling is playing an increasingly paramount role in providing quantitative insight into multiple fields [4]. It has contributed to a better realization of the mechanisms of various chronic diseases and infectious diseases [5]. For instance, currently, we can see extensive use of mathematical modeling in understanding the mysterious mechanisms of ongoing highly infectious disease COVID-19. It has also availed understanding of the mechanisms of various critical phenomena, such as wound healing, morphogenesis, and blood-cell production. It has received increasing attention because modeling and simulation allow rapid, cost-effective testing and formulation of novel hypotheses [6]. Investigation of the natural phenomena and various effects of climate change is another major field of mathematical modeling [7]. Due to globalization and the diversity of living objects, climate change has been a pivotal aspect of research over the years [8–10]. Mathematical modeling plays a pivotal role in earth science-related aspects in various branches of environmental sciences. It may enhance the solution to the catastrophic incidents and adversities of unplanned global biodiversity and reduce the threats of the severe pollution caused over the decades. Artificial intelligence is vital for treating unwanted climate changes with long-term natural effects [11]. Mathematical modeling is the fundamental base of modern computing science that enhances the incorporation of biological models with artificial intelligence [12]. So, mathematical modeling can be used to improve prognosis, management, and control strategies for diseases. Also, properly utilizing mathematical modeling in the environmental sciences, especially in the remedy of climate changes, proper time management, and optimization of several costs, can be ensured [13].

We are aiming for computer-based simulation through the Python platform, where Age of Information (AoI) plays a prominent role [14]. For the quantitative approaches to data prediction, real-time data is the pivot aspect. In forecasting for the future or data prediction methods, the data attained from past periods enhance the logical assumption of the next phenomena. The majority of the data prediction tools use the primary data that must be acquired from trustworthy sources in an impartial manner [15]. Data-driven prediction models are mostly applied for the forecasting of pandemic situations. Data collection, classification, model generation, and validity testing are very closely connected to the AoI [16]. In those sequences of activities, AoI justifies data modernity by investigating the requirement of the proposed model, which also ensures the usefulness and successive updates of the information over the required period [17]. In the present days, optimization of the data prediction accuracy is another prime concern of the AoI [18]. Data feasibility, adjustment to the proposed models, and analysis of the physical attributes greatly rely on AoI-based strategies [19]. For the betterment of the data collection, transmission, allocation, and implementation Internet of Things (IoT) act as the key supporting mechanism [20, 21]. Sensor-based artificial intelligence (AI) with remote access is a distinguished ingredient of IoT that makes the remote sensing data arrangement more feasible than in the past [22]. Machine learning (ML) technologies provide a wide range of facilities for data structure, similarity analysis, and prediction yielding maximum efficiency with minimum effort [23]. Presently, IoT is massively used for healthcare functions, basically for decision-making features. In the current COVID-19 spreading, the overall scenario of community transmission, deaths, recoveries, and medication information is accommodated through the various modes of IoT [24, 25].

Epidemiological modeling is done by integrating mathematical modeling into the system that works on a certain population, which can be divided into nonintersecting classes, such as susceptible (*S*(*t*)), infective (*I*(*t*)), and removed (*R*(*t*)) [26, 27]. Infective classes of the population and then specify the behavior of casual agents in different compartments were analyzed over time [28, 29]. The simplest compartmental model is SIR, which is used for epidemiological modeling [30]. Since each disease is distinct, models must be adjusted depending on the epidemic's parameters and components. SIS, SIR, SIRD, SEIR, SIQR, and SEIRD are some of the extended versions of SIR that researchers use for epidemiological modeling [31–33]. Using epidemiological models, we can show how different public health interventions may affect the outcome of the epidemics [34, 35].

Epidemiological modeling is a great tool for estimating the future of a pandemic, and researchers always try to optimize these models. Great work to comprehend these models has been proposed by Herbert Hethcote, in which he presented overviews of different compartmental models and their theoretical characteristics [36]. Jesus Fernandez-Villaverde and Charles I. Jones have introduced the SIRD model to estimate standard epidemiological modeling of COVID-19 [37]. However, only death data from many countries around the world was used in their models. They have made certain additions, including inverting the SIRD model and introducing an additional recovery state for those who seem to be infectious for a couple of days but took longer to recover. Through the simulation, they tried to predict the possible outcomes of COVID-19. Saulo B. Bastos and Daniel O. Cajueiro have also used compartmental models such as SIR, SIRD, and SIRED to forecast the growth of COVID-19 in Brazil [38]. They proposed two variations of the SIR model and added a parameter to analyze the effect of social distancing. However, an optimal control method for models like SIR, SIRD, and SEIRD can be found in the work of Morton and Wickwire [39].

The main challenge in epidemiological modeling is finding accurate data on cases. So researchers have to make some assumptions for the sake of their work. Since many parameters get ignored this way, the accuracy level significantly fluctuates. Fernandez-Villaverde and Charles I. Jones had faced similar kinds of difficulties [37]. As they have only focused on death data, they came to a conclusion based on a relatively simple model. Then again, as the massive test campaign did not take place, the exact number of deaths is still unsure. Saulo B. Bastos, in his paper, has urged to test the population as there is a possibility that an asymptomatic individual too can be a carrier of the virus [38].

To fight against any disease, we need to know the exact number of people at high risk and provide them with the proper healthcare. However, it is hard to do in such overcrowded countries as Bangladesh, India, and Indonesia. As a result, a great number of people remain uncovered (those who are susceptible to the coronavirus but are not tested). Some components are accountable for this, for instance, insufficient funding for running a massive campaign, hurriedly collecting data, and lacking human resources to reach every corner of the country. Similarly, due to social and monetary issues, a significant number of apathetic people (those who are unwilling to take a test or maintain proper instructions after being exposed) intend to refrain from healthcare activities. Most apathetic people are illiterate and make their decision over some rumor. So they fear going through the testing procedure. Another main reason is that they cannot manage enough money on time to go to the hospital and receive treatment.

The SEIRD model, one of the epidemiological models that researchers and epidemiologists use to predict the future of a pandemic, comprises five branches, namely, susceptible (*S*), exposed (*E*), infected (*I*), recovered (*R*), and dead (*D*) [40]. Susceptible are those groups of people who are not infected but are at high risk of getting COVID-19. Those who are prone to the infection can be categorized as exposed. The infected category is for those who have tested COVID-19 positive. Finally, after these three states, people would either recover or die. The basic SEIRD model is shown in Figure 1.

We have added two more branches to the main SEIRD model in our work, namely, uncovered (*U*) and apathetic (*A*), intending to estimate the future of COVID-19. This uncovered stage is a subcategory of susceptible, which means some people remain uncovered even if they are at high risk, and the apathetic people are included in the exposed state who does not receive the proper treatment. In this work, we have utilized real-time input-data-based simulation techniques incorporating Python programming with the mathematical induction approach. Our system is designed and trained to take the input data and provide the predicted data with significant accuracy. We have justified the proposed model by comparing the predicted data with the real-time data by the graphical manifestation. Error analysis of the data prediction is provided through the relative error expressed as the percentage, where the figurative interpretation is incorporated with the statistical analysis. Finally, some numerical assessment was done by the correlation and regression analysis. We expect this work will facilitate exploring the spreading characteristics of COVID-19, along with its future growth. It may help in making different government policies as well.

## 2. Materials and Methods

Presently, COVID-19 is one of the atrocious epidemics in the world. From a statistical point of view, the SEIRD model is being studied systematically. Too many researchers have proposed various models using this, as we mentioned before. Similarly, we have investigated the extensions of the basic SEIRD model in our previous work and introduced two extended models by adding the branches uncovered and apathetic, respectively [41]. The extended SEIRD models are exhibited below in subfigures of Figure 2, respectively.

List of the parameters with the corresponding symbols are given in Table 1.

Later on, it seemed that if the whole ingredients could be shown in a single model rather than separate models, the acceptability and adaptability of this updated SEIRD model would be preferable to before. Consequently, we are proposing an improved version of the SEIRD model, where we have merged the previous extensions.

### 2.1. Proposed Model

In the proposed model, we are incorporating the basic components of the SEIRD model with that of the unprivileged classes of the population, namely, the uncovered and apathetic. The improved proposed version of the extended SEIRD model would be able to illustrate the real-time scenario of the pandemic situation in Third World countries. The proposed extension of the SEIRD model is depicted in Figure 3.

### 2.2. Mathematical Formulation

The components connected to the physical phenomena incorporated with the logical affirmation enhance the composition of a mathematical model that can comprehensively manifest the attributes of the objective population. The following system of governing equations designs the formulation of the proposed improved epidemiological model.

(1) $$\begin{array}{c} ∆S=-\alpha \frac{S\times E}{N}-\beta \frac{S\times U}{N}, \end{array}$$

(2) $$\begin{array}{c} ∆U=\beta \frac{S\times U}{N}-\sigma U-\tau \;U, \end{array}$$

(3) $$\begin{array}{c} ∆E=\alpha \frac{S\times E}{N}-\gamma I-\lambda A-\rho I_{s}, \end{array}$$

(4) $$\begin{array}{c} ∆A=\lambda A-\omega A-\eta A, \end{array}$$

(5) $$\begin{array}{c} ∆I=\gamma I-\delta I-\mu I, \end{array}$$

(6) $$\begin{array}{c} ∆I_{s}=\rho I_{s} \end{array}$$

(7) $$\begin{array}{c} ∆D_{I}=\delta I, \end{array}$$

(8) $$\begin{array}{c} ∆R_{I}=\mu I, \end{array}$$

(9) $$\begin{array}{c} ∆D_{A}=\omega A, \end{array}$$

(10) $$\begin{array}{c} ∆R_{A}=\eta A, \end{array}$$

(11) $$\begin{array}{c} ∆D_{U}=\sigma U, \end{array}$$

(12) $$\begin{array}{c} ∆R_{U}=\tau \;U. \end{array}$$

Variations of the different components of the epidemiological models are contingent on the rate parameters of the governing equations. Equations (1) to (12) are expressing the successive increment in the desired components of the proposed model. In each equation, the target component is taken as the node, whereas incoming and outgoing components are taken as the positive and negative flows for the corresponding component. Rate parameters are taken as the weight for each incoming and outgoing component. The linear combinations of the total flows provide the desired increment of the target component.

To find the rate parameters of the proposed model, we have to solve the Equations (1) to (12). The simplified forms of those rate parameters are given below.

(13) $$\begin{array}{c} \tau =\frac{∆R_{U}}{U}, \end{array}$$

(14) $$\begin{array}{c} \sigma =\frac{∆D_{U}}{U}, \end{array}$$

(15) $$\begin{array}{c} \eta =\frac{∆R_{A}\;}{A}, \end{array}$$

(16) $$\begin{array}{c} \omega =\frac{∆D_{A}}{A}, \end{array}$$

(17) $$\begin{array}{c} \mu =\frac{∆R_{I}\;}{I}, \end{array}$$

(18) $$\begin{array}{c} \delta =\frac{∆D_{I}\;}{I}, \end{array}$$

(19) $$\begin{array}{c} \rho =\frac{∆I_{s}}{I_{s}}, \end{array}$$

(20) $$\begin{array}{c} \gamma =\frac{∆I+∆D_{I}+∆R_{I}\;}{A}, \end{array}$$

(21) $$\begin{array}{c} \lambda =\frac{∆A+∆D_{A}+∆R_{A}\;}{A}, \end{array}$$

(22) $$\begin{array}{c} \beta =\frac{∆U+∆D_{U}+∆R_{U}}{S\times U}\times N, \end{array}$$

(23) $$\begin{array}{c} \alpha =\frac{∆E+∆I+∆D_{I}+∆R_{I}+∆A+∆D_{A}+∆D_{A}+∆I_{s}}{S\times E}\times N. \end{array}$$

## 3. Results and Discussions

Validation of the proposed model is investigated in this section with practical pieces of evidence. We have applied the improved SEIRD model to analyze and forecast the COVID-19 circumstances in Bangladesh. We have observed the individuals of the cases for the components susceptible, exposed, uncovered, isolated, infected, and apathetic, along with the occurrences of deaths and recoveries. In this scheme of investigation, we have used the experimental data collected from some trustworthy sources and configured them according to the requirement of the proposed model.

### 3.1. Data Collection Scheme and Setting Arrangement

A well-grounded data set is a fundamental prerequisite for validating mathematical models. The present work scrutinizes a very sophisticated contemporary issue, namely, COVID-19. Thus, the selection of a real-time data set is a very crucial task. Attaining authentic data is always a cumbersome assignment. In the data collection process, we have inquired into several types of public data sources, for instance, health-care-related national and international news portals, and open-source data directories of government and nongovernment agencies. We have collected the COVID-19-related information from social sites as well. Moreover, due to their absence in well-established institutions, few data are collected locally from newspapers and news bulletins.

The assembled data set comprised the columns of the total number of susceptible, exposed, uncovered, isolated, infected, and apathetic cases with corresponding deaths and recoveries. Here, we can refer some reliable sources of practical data, such as DGHS Bangladesh, Corona Info, IEDCR, Worldometer, and WHO. The real-time data of 46 days from 16 June 2021 to 31 July 2021 are collected and considered in this research for predicting the data for desired upcoming days.

### 3.2. Methodology of the Data Prediction

The desired prediction will be estimated by the proposed model utilizing numerical simulations. The Python programming language will be assimilated for the simulation codes. To predict the future data, from the previous works, it has been seen that the SEIRD models can be trained for at most 7 days, and it has been extended to 15 days in [41]. Now, we aim to assign the proposed model for training over more than 15 days to predict the future data for longer. We employed the real-time data for 21 days from 11 July 2021 to 31 July 2021 and predicted the future data for 30 days from 1 August 2021 to 30 August 2021. According to the successive prediction process, the proposed model learns the data every 30 days, predicts the outcome of the next day, and does the same for the next days, which is a recurrence prediction strategy.

### 3.3. Figurative Comparison of the Predicted Data with the Real-Time Data

To justify the validity and accuracy of the proposed model, a figurative comparison between real-time data and the predicted data for the target components is considered. Predictions of the total number of cases are pointed out for each component, and the number of individual cases can be found by taking successive differences of two consecutive days.

Figures 4, 5, and 6 demonstrate the comparison of real-time data and predicted data of the total number of uncovered, infected, and apathetic cases along with the corresponding deaths and recoveries, respectively.

Figures 7 and 8 exhibit the comparison of the real-time and predicted data of the total number of exposed and isolated cases. The dates of the target period are depicted in *x* axis, whereas the number of respective cases is depicted in *y* axis. Scaling of *y* axis is distinctly taken so that the difference between real-time and predicted data could be significantly ascertained.

The subfigures of Figures 4, 5, and 6 illustrate admissible resemblance of the real-time and predicted data of uncovered, infected, and apathetic cases along with the corresponding deaths and recoveries, respectively. The prediction process was excellent for about 20 days, and then, the deviation started for a few cases. However, this is not surprising as the real-time data pattern was nonlinear, whereas in most of the cases, the pattern of predicted data lost the nonlinearity.

From Figures 7 and 8, it is conspicuous that both the real-time and predicted data for the exposed and isolated cases have nonlinearity. Still, the trend is not the same and has noticeable fluctuations. This happened due to the lack of trustworthiness of the collected data and peoples' unwillingness to maintain public health regulations. Moreover, many of the exposed and isolated cases were not firmly recorded because of the initial infrastructural infelicity of the healthcare institutions.

Thus, from the figurative comparison, it can be claimed that the proposed model can be competently used to predict the future data for the epidemics for up to 20 days for most of the components and almost 30 days for some of the components.

It can be said that, if we reduce the number of prediction days, the fluctuations between the real-time data and predicted data for the target cases can be optimized. Also, if we can get more reliable open-source real-time data, the better predictions can be gained by utilizing the proposed model.

### 3.4. Error Analysis

Since we have scaled the graphs for exploring the variations of the real-time and predicted data distinguishable, the scales were not uniform for all of the components of the epidemiology. So, to clarify the variations properly, their descriptive analysis is essential. The relative errors for the target components expressed in percentage are appraised in the error analysis.  Figure 9 displays the relative errors in percentage for all the components for 30 days from 1 August 2021 to 30 August 2021.

From Figure 9, it is obvious that for the first 10 days, no significant errors can be seen for all the components but in isolation. The errors for all components other than isolation are allowable for up to the next 10 days. For the final 10 days, the errors for *D*_*I*_, *R*_*I*_, and *E* are comparatively significant, whereas the error for *I*_*s*_ is remarkable. The unbounded error for isolation cases is due to the improper healthcare management and ignorance of the basic healthcare regulations of the mass people in practical, which are methodically neglected in the prediction process. To disclose the plenary scenario of the error analysis, a tabular exposure of the statistical ingredients of error analysis, including minimum value, maximum value, average, and standard deviation (SD) of the relative errors, is provided in Table 2.

So, from the graphical and tabular pieces of evidence, it is ascertained that almost all of the target components of the epidemiology proposed model can be suitably implemented.

### 3.5. Correlation and Regression Analysis

The number of deaths and recoveries are the most prominent components of the epidemics, and most epidemiological models are designed to predict them essentially. From the previous sections, it is already justified that the component's deaths and recoveries can be properly predicted by implementing the proposed model. In this section, the correlation and regression analysis of the real-time and predicted data will be done for the deaths and recoveries of the uncovered, infected, and apathetic cases, respectively.

Table 3 displays the correlation coefficients of the deaths and recoveries of several cases' real-time and predicted data. The table shows that the deaths and recoveries of those cases are perfectly correlated with a correlation coefficient of almost 1. However, according to the numerical evidence, predicted data shows a better correlation than real-time data.

Table 4 displays the regression coefficients of the deaths and recoveries of several cases' real-time and predicted data. From the table, it is seen that for both the real-time and predicted data, the number of deaths is dominant over the number of recoveries. In all cases, the rate of the dominance of the number of deaths is a bit higher for the predicted than that of the real-time data.

It is crucial to predict the number of deaths and recoveries according to the cases arising from uncovered, infected, and apathetic people. The regression lines for predicting future data of deaths and recoveries depending on the current data of the uncovered, infected, and apathetic cases for both real-time and predicted data are given below.

(24) $$\begin{array}{c} {\hat{D}}_{U}^{\left(\text{real}\right)}=-933.6246+0.0273U^{\left(\text{rea}l\right)}, \end{array}$$

(25) $$\begin{array}{c} {\hat{R}}_{U}^{\left(\text{real}\right)}=-8909.3481+0.6215U^{\left(\text{real}\right)}, \end{array}$$

(26) $$\begin{array}{c} {\hat{D}}_{I}^{\left(\text{real}\right)}=-10049.5275+0.0241I^{\left(\text{real}\right)}, \end{array}$$

(27) $$\begin{array}{c} {\hat{R}}_{I}^{\left(\text{real}\right)}=-758521.1255+1.4507I^{\left(\text{real}\right)}, \end{array}$$

(28) $$\begin{array}{c} {\hat{D}}_{A}^{\left(\text{real}\right)}=-3943.1641+0.0303A^{\left(\text{real}\right)}, \end{array}$$

(29) $$\begin{array}{c} {\hat{R}}_{A}^{\left(\text{real}\right)}=-43714.3876+0.6484A^{\left(\text{real}\right)}, \end{array}$$

(30) $$\begin{array}{c} {\hat{D}}_{U}^{\left(\text{predicted}\right)}=-4804.5386+0.0346U^{\left(\text{predicted}\right)}, \end{array}$$

(31) $$\begin{array}{c} {\hat{R}}_{U}^{\left(\text{predicted}\right)}=-111093.6636+0.8149U^{\left(\text{predicted}\right)}, \end{array}$$

(32) $$\begin{array}{c} {\hat{D}}_{I}^{\left(\text{predicted}\right)}=-7768.5885+0.0226I^{\left(\text{predicted}\right)}, \end{array}$$

(33) $$\begin{array}{c} {\hat{R}}_{I}^{\left(\text{predicted}\right)}=-791304.2687+1.4961I^{\left(\text{predicted}\right)}, \end{array}$$

(34) $$\begin{array}{c} {\hat{D}}_{A}^{\left(\text{predicted}\right)}=-14401.8629+0.0451A^{\left(\text{predicted}\right)}, \end{array}$$

(35) $$\begin{array}{c} {\hat{R}}_{A}^{\left(\text{predicted}\right)}=-348195.9455+1.0813A^{\left(\text{predicted}\right)}. \end{array}$$

So, by exerting the number of uncovered, infected, and apathetic cases in the above regression lines, the number of future deaths and recoveries corresponding to these cases can be suitably predicted.

## 4. Conclusion

In this work, an improved SEIRD model was derived and applied for the underprivileged people in the contemporary pandemic, a combination of two extensions of the basic SEIRD model derived in previous work. The uncovered and apathetic cases and the associated deaths and recoveries are constituted in this improved version of the SEIRD model. As the data-driven validation of the proposed model, we explored the pervasiveness of COVID-19 from the Bangladesh perspective. Implementing the improved SEIRD model, we have gained the appeasement outcomes in all components except the isolated cases. The reasons behind the infirmity of predicting isolated cases are conferred. From the figurative comparison and analysis of error, it is apparent that the improved SEIRD model can practically implant for the prediction of future data based on the real-time data. From the statistical overview delineated in this work, it can be said that the deaths and recoveries are perfectly correlated for all sorts of real-time data cases, and the predicted data follows the same trend. According to the regression analysis, it is evident that the number of deaths is expressly over the number of recoveries for both real-time and predicted data. The regression lines for predicting future deaths and recoveries according to the uncovered, infected, and apathetic cases are also formed. From both the real-time and predicted data, it is comprehensible that though the numbers of uncovered and apathetic cases are not negligible, in contrast to the infected cases, these cases are enough diminutive. Also, the number of recoveries appreciably outplayed the number of deaths on every occasion.

The number of uncovered cases increased due to the lack of skilled healthcare workers, misconceived authorities, and impractical infrastructure. Since the percentage of deaths is significantly more contemptible than the percentage of recoveries, which raised the apathetic cases among the uneducated and troublesome people. Socio-economic conditions and deficiency of epidemiological knowledge are also responsible for escalating the apathetic cases.

Recently, a novel epidemiological disease, Monkeypox, evolved and propagated in many countries. The next research will try implementing the improved SEIRD model for Monkeypox. A machine learning algorithm will be derived to support the improved SEIRD model, and it is expected that the machine learning approach will resolve the issue that occurred in isolated cases.

## Figures and Tables

**Figure 1:** Basic SEIRD model.

**Figure 2:** Flowcharts of the models designed in [41].

**Figure 3:** Flowchart of the improved SEIRD model.

**Figure 4:** Comparison of the real-time data and predicted data for the uncovered population with respective deaths and recoveries.

**Figure 5:** Comparison of the real-time data and predicted data for the infected population with respective deaths and recoveries.

**Figure 6:** Comparison of the real-time data and predicted data for the apathetic population with respective deaths and recoveries.

**Figure 7:** Comparison of the real-time data and predicted data for the exposed population.

**Figure 8:** Comparison of the real-time data and predicted data for the isolated population.

**Figure 9:** Relative errors of the data prediction for the target components.

**Table 1:** List of parameters.

Symbol	Name of the parameter
*N*	Total population
*S*	Susceptible population
*E*	Exposed population
*I*	Infected population
*D*_*I*_	Died population from infection
*R*_*I*_	Recovered population from infection
*I*_*s*_	Isolated population
*U*	Uncovered population
*D*_*U*_	Died population from uncovered
*R*_*U*_	Recovered population from uncovered
*A*	Apathetic population
*D*_*A*_	Died population from apathetic
*R*_*A*_	Recovered population from apathetic
*α*	Rate of exposed population
*β*	Rate of uncovered population
*λ*	Rate of apathetic population
*ρ*	Rate of isolated population
*γ*	Rate of infected population
*δ*	Rate of infected population death
*μ*	Rate of infected population recovery
*σ*	Rate of uncovered population death
*τ*	Rate of uncovered population recovery
*ω*	Rate of apathetic population death
*η*	Rate of apathetic population recovery

**Table 2:** Error analysis of the data prediction.

Component	Minimum value of RE (%)	Maximum value of RE (%)	Average of RE (%)	SD of RE (%)
*U*	0.019989619	1.333720125	0.699549631	0.388538502
*D*_*U*_	0.029713267	4.402515723	1.166717887	1.243956252
*R*_*U*_	0.004975998	4.924759094	1.308852504	1.452518706
*E*	0.137083351	5.928316544	3.103290897	1.729532422
*I*_*s*_	2.223648509	31.8528292	13.06339325	9.295056472
*I*	0.064410718	5.380764019	1.623503267	1.386483902
*D*_*I*_	0.021138968	7.219343696	1.898730126	2.118184882
*R*_*I*_	0.313575063	10.37146118	3.301024967	3.066394265
*A*	0.063733904	4.188094412	3.048232455	1.277145975
*D*_*A*_	0.097092092	2.076857869	0.832487017	0.514673584
*R*_*A*_	0.017224001	2.571790272	0.655207578	0.689055442

**Table 3:** Correlation coefficients of the number of deaths and recoveries for different categories of the population.

Category	Uncovered	Infected	Apathetic
Real-time data	0.99997024	0.99957924	0.99926613
Predicted data	0.99999994	0.99999998	0.99999996

**Table 4:** Regression coefficients of the number of deaths and recoveries for different categories of the population.

Category	Uncovered		Infected		Apathetic	
Dominance	*D*_*U*_	*R*_*U*_	*D*_*I*_	*R*_*I*_	*D*_*A*_	*R*_*A*_
Real-time data	22.7440	0.0440	60.2672	0.0166	21.7049	0.0460
Predicted data	23.5270	0.0425	66.1188	0.0151	23.9799	0.0417

## Data Availability

Data can be found at https://github.com/mu2mahmud/Improved-epidemiological-model/.

## References

[1] Bailey J. E. (1998). Mathematical modeling and analysis in biochemical engineering: past accomplishments and future opportunities. *Biotechnology Progress*.

[2] Kermack W. O., McKendrick A. G. (1927). A contribution to the mathematical theory of epidemics. *Proceedings of the Royal society of london. Series A, Containing papers of a mathematical and physical character*.

[3] Costa A., Pires M., Resque R., Almeida S. (2021). Mathematical modeling of the infectious diseases: key concepts and applications. *Journal of Infectious Diseases and Epidemiology*.

[4] Karplus W. J. (1977). The spectrum of mathematical modeling and systems simulation. *ACM SIGSIM Simulation Digest*.

[5] Zaman G., Jung I. H., Torres D. F., Zeb A. (2017). Mathematical modeling and control of infectious diseases. *Computational and Mathematical Methods in Medicine*.

[6] Bhaskar S., Sinha A., Banach M. (2020). Cytokine storm in COVID-19—immunopathological mechanisms, clinical considerations, and therapeutic approaches: the reprogram consortium position paper. *Frontiers in Immunology*.

[7] Eikenberry S. E., Gumel A. B. (2018). Mathematical modeling of climate change and malaria transmission dynamics: a historical review. *Journal of Mathematical Biology*.

[8] Young O. R., Berkhout F., Gallopin G. C., Janssen M. A., Ostrom E., Van der Leeuw S. (2006). The globalization of socio-ecological systems: an agenda for scientific research. *Global Environmental Change*.

[9] Eriksen T. H. (2020). *Globalization: The Key Concepts*.

[10] Moser S. C. (2010). Communicating climate change: history, challenges, process and future directions. *Wiley Interdisciplinary Reviews: Climate Change*.

[11] Rodriguez-Delgado C., Bergillos R. J. (2021). Wave energy assessment under climate change through artificial intelligence. *Science of the Total Environment*.

[12] Levin S. A., Grenfell B., Hastings A., Perelson A. S. (1997). Mathematical and computational challenges in population biology and ecosystems science. *Science*.

[13] Meerschaert M. M. (2013). *Mathematical Modeling*.

[14] Yates R. D., Kaul S. K. (2018). The age of information: real-time status updating by multiple sources. *IEEE Transactions on Information Theory*.

[15] Hua J., Shaw R. (2020). Corona virus (covid-19)“infodemic” and emerging issues through a data lens: the case of China. *International journal of environmental research and public health*.

[16] Wong Z. S., Zhou J., Zhang Q. (2019). Artificial intelligence for infectious disease big data analytics. *Infection, disease & health*.

[17] Zens M., Brammertz A., Herpich J., Südkamp N., Hinterseer M. (2020). App-based tracking of self-reported COVID-19 symptoms: analysis of questionnaire data. *Journal of medical Internet research*.

[18] Chakraborty T., Ghosh I. (2020). Real-time forecasts and risk assessment of novel coronavirus (COVID-19) cases: a data-driven analysis. *Chaos, Solitons & Fractals*.

[19] Tuli S., Tuli S., Tuli R., Gill S. S. (2020). Predicting the growth and trend of COVID-19 pandemic using machine learning and cloud computing. *Internet of Things*.

[20] Yerpude S., Singhal T. K. (2017). Impact of internet of things (IoT) data on demand forecasting. *Indian Journal of Science and Technology*.

[21] Abd-Elmagid M. A., Pappas N., Dhillon H. S. (2019). On the role of age of information in the internet of things. *IEEE Communications Magazine*.

[22] Quer G., Radin J. M., Gadaleta M. (2021). Wearable sensor data and self-reported symptoms for COVID-19 detection. *Nature Medicine*.

[23] Thielen N., Werner D., Schmidt K., Seidel R., Reinhardt A., Franke J. A machine learning based approach to detect false calls in SMT manufacturing.

[24] Javaid M., Khan I. H. (2021). Internet of things (IoT) enabled healthcare helps to take the challenges of COVID-19 pandemic. *Journal of Oral Biology and Craniofacial Research*.

[25] Sultana N., Tamanna M. (2021). Exploring the benefits and challenges of internet of things (IoT) during COVID-19: a case study of Bangladesh. *Discover Internet of Things*.

[26] Cooper I., Mondal A., Antonopoulos C. G. (2020). A SIR model assumption for the spread of COVID-19 in different communities. *Chaos, Solitons & Fractals*.

[27] Okabe Y., Shudo A. (2020). A mathematical model of epidemics—a tutorial for students. *Mathematics*.

[28] Sattenspiel L. (1990). Modeling the spread of infectious disease in human populations. *American Journal of Physical Anthropology*.

[29] Tiwari A. (2020). Modelling and analysis of COVID-19 epidemic in India. *Journal of Safety Science and Resilience*.

[30] Rodrigues H. S. (2016). Application of SIR epidemiological model: new trends. https://arxiv.org/abs/1611.02565.

[31] Nesteruk I. (2020). SIR-simulation of corona pandemic dynamics in Europe. https://www.medrxiv.org/content/10.1101/2020.04.22.20075135v1.

[32] Biswas K., Khaleque A., Sen P. (2020). COVID-19 spread: reproduction of data and prediction using a SIR model on Euclidean network. https://arxiv.org/abs/2003.07063.

[33] Rˇadulescu A., Williams C., Cavanagh K. (2020). Management strategies in a SEIR-type model of COVID-19 community spread. *Scientific Reports*.

[34] Canzani E., Lechner U. (2015). *Insights from modeling epidemics of infectious diseases-a literature review*.

[35] Garner M., Hamilton S. (2011). Principles of epidemiological modelling. *Revue Scientifique et Technique-OIE*.

[36] Hethcote H., Zhien M., Shengbing L. (2002). Effects of quarantine in six endemic models for infectious diseases. *Mathematical Biosciences*.

[37] Fernández-Villaverde J., Jones C. I. (2020). *Estimating and simulating a SIRD model of COVID-19 for many countries, states. and cities*.

[38] Bastos S. B., Cajueiro D. O. (2020). Modeling and forecasting the early evolution of the COVID-19 pandemic in Brazil. *Scientific Reports*.

[39] Morton R., Wickwire K. H. (1974). On the optimal control of a deterministic epidemic. *Advances in Applied Probability*.

[40] Fonseca i Casas P., García i Carrasco V., Garcia i Subirana J. (2020). SEIRD COVID-19 formal characterization and model comparison validation. *Applied Sciences*.

[41] Mugdha S. B., Uddin M., Islam M. (2021). Extended epidemiological models for weak economic region: Case studies of the spreading of COVID-19 in the South Asian subcontinental countries. *BioMed Research International*.

